# Recent Preclinical Insights Into the Treatment of Chronic Traumatic Encephalopathy

**DOI:** 10.3389/fnins.2020.00616

**Published:** 2020-07-07

**Authors:** Patrick W. Breen, Vaishnav Krishnan

**Affiliations:** ^1^Department of BioSciences, Rice University, Houston, TX, United States; ^2^Department of Neurology, Baylor College of Medicine, Houston, TX United States

**Keywords:** chronic traumatic encephalopathy, tauopathy, neurodegeneration, traumatic brain injury, neuroinflammation

## Abstract

Chronic traumatic encephalopathy (CTE) is a neurodegenerative condition associated with significant mortality and morbidity. The central pathophysiological mechanisms by which repetitive cranial injury results in the neurodegeneration of CTE are poorly understood. Current well-established working models emphasize a central role for trauma-induced excessive phosphorylation and accumulation of insoluble tangles of Tau protein. In this review, we summarize recent data from preclinical animal models of CTE where a series of candidate treatments have been carefully evaluated, including kinase inhibitors, antibody therapy, and anti-inflammatory therapies. We discuss the overall translational potential of these approaches and provide recommendations for future bench-to-bedside treatment strategies.

## Introduction

Chronic traumatic encephalopathy (CTE) is a neurodegenerative brain disease caused by the cumulative impact of repetitive mild traumatic brain injury (rmTBI). Initial symptoms manifest as non-specific cognitive and neuropsychiatric impairments, including depression and heightened aggression, and eventually progress to include a variety of motor impairments and cognitive decline (Montenigro et al., 2014). While this syndrome has been appreciated for more than a century by many terms (e.g., “punch-drunk syndrome” or *dementia pugilistica*) (Martland, 1928), it has recently been recognized formally as CTE by both the media and the scientific community. Individuals at highest risk include subjects playing contact sports such as football, boxing, and soccer. Athletes participating in American football are at a particularly high risk; NFL (National Football League) players develop CTE-related dementia at five times the rate of age-matched controls (Stein et al., 2014). In a recent study, up to 87% of postmortem brain samples donated by NFL players displayed pathological evidence of CTE, and histological markers of CTE severity varied proportionally with years of football played (Mez et al., 2020). Military personnel with repetitive blast exposures are also at risk of developing CTE (Goldstein et al., 2012). Aside from supportive treatment designed to address specific symptoms (such as depression or comorbid seizures), there are no specific disease modifying treatments or reliable *in vivo* diagnostic markers for individuals with suspected CTE (Stein et al., 2014).

## Comorbidities and Neuropathology

The initial symptoms of CTE may not occur until years or even decades after rmTBI and may affect cognitive and/or emotional domains. By one classification system, symptoms occurring in more than 50% of “mild” CTE (Stages 1 or 2) include impulsivity, depression, physical and verbal violence, memory loss, and suicidality. Severe CTE (Stages 3 or 4) is characterized by additional symptoms such as language impairments, visuospatial deficits, parkinsonism, and dementia-like deficits (Mez et al., 2017). CTE is often comorbid with other neurological conditions including Lewy body disease (LBD) (Adams et al., 2018), amyotrophic lateral sclerosis (ALS) (Walt et al., 2018), and occasionally primary prionopathies (Nemani et al., 2018). Given the clinical heterogeneity of CTE, appropriate diagnostic criteria are still a subject of debate. For example, another proposed classification system divides CTE syndromes into four distinct subtypes: behavioral/mood variant, cognitive variant, mixed variant, and dementia (Montenigro et al., 2014).

While there remain many unknowns about the molecular and cellular pathological changes that are presumably incited by repeated cranial impact, a strong consensus has unified around the pathophysiological role of hyperphosphorylated tau (“p-tau”) accumulation and neurofibrillary tangle (NFT) formation (McAteer et al., 2017). Thus, CTE falls into a family of neurodegenerative diseases known as tauopathies (Noble et al., 2013) which includes Alzheimer’s disease (AD), frontotemporal lobar degeneration (FTLD, previously known as Pick’s disease), and progressive supranuclear palsy (PSP). Accumulations of hyperphosphorylated tau have been linked to cytoskeletal dysfunction, DNA damage, and synaptic dysfunction (Noble et al., 2013), although abnormal increases in dephosphorylated tau may also contribute to CTE pathology (Rubenstein et al., 2019). Other biomarkers that have been documented in patients with CTE include increases in beta-amyloid, neuron-specific enolase (NSE), and glial fibrillary-associated protein (GFAP) (McKee et al., 2016). A formal postmortem diagnosis of CTE requires the identification of perivascularly accumulated p-tau neurofibrillary tangles (NFTs) at sulcal depths in the cerebral cortex. These can be graded into four levels of severity based on the extent of atrophy and NFT accumulation (McKee et al., 2015). While gross neurological abnormalities are generally not present early in the disease, late stage CTE brains (Figure 1) can display gross white and gray matter atrophy accompanied by ex vacuo ventricular dilatation (McKee et al., 2016).

**FIGURE 1:** Coronal slices of advanced CTE **(A)** compared to a normal brain **(B)**. CTE brain shows enlargement of the ventricles (1–2), septum pellucidum (3), medial temporal lobe (4), and mammillary bodies (5) (Stern et al., 2011). Permission obtained from John Wiley and Sons through PM&R Journal. License #: 4730951503528.

While postmortem analysis remains the standard for CTE diagnosis, current research has focused on finding reliable *in vivo* premortem diagnostic markers. In particular, PET imaging with radiotracers such as [F-18]FDDNP (which binds insoluble protein aggregates) has been used to identify tau and beta-amyloid patterns consistent with CTE (Barrio et al., 2015). One challenge to reliably diagnosing CTE is its pathophysiological similarity to other tauopathies. However, not all tauopathies are molecularly similarly: Tau has six isoforms, and in contrast to tauopathies like FTLD and PSP, only CTE and AD pathophysiology involve all six tau isoforms (Katsumoto et al., 2019).

The relationship between Alzheimer’s disease (AD) and CTE remains somewhat enigmatic. Both tauopathies share a series of culprit tau phosphorylation sites (Katsumoto et al., 2019) and TBI (but not necessarily rmTBI) is a risk factor for AD (Nemetz et al., 1999; Schaffert et al., 2018). Additionally, a mixed CTE/AD phenotype has been reported (Kanaan et al., 2016), leading some researchers to question whether CTE can eventually lead to AD (Katsumoto et al., 2019). Nevertheless, at a cellular and histological level, AD and CTE are considered distinct tauopathies. AD typically results in diffuse brain atrophy and extensive Aβ pathology, whereas CTE typically yields perivascular tau agglomeration in the ventricles and frontal lobe, primarily at sulcal depths (Turner et al., 2016). P-tau pathology in CTE contrasts from that in AD by preferentially affecting superficial layers (II–III) and hippocampal regions CA2 and CA4 (McKee et al., 2016). Clinically, AD results in a more gradual cognitive deterioration characterized by prominent memory impairment, whereas in CTE, mood and emotional symptoms may be more conspicuous, particularly in early-onset CTE (Stern et al., 2011; Turner et al., 2016).

Given the major knowledge gaps in our understanding of CTE pathogenesis, as well as limitations in available premortem diagnostic biomarkers, it is not surprising that there are currently no ongoing clinical trials for the treatment of CTE. However, in light of the proposed pathophysiological overlaps between AD and CTE, several therapies that have demonstrated preclinical success in AD models have now been applied to CTE models. This review summarizes key recent findings within this body of literature which have focused on accumulations of hyperphosphorylated tau aggregates as both a direct mediator of neuronal injury and a histological biomarker of disease severity.

## Animal Models and Methodology

By definition, the vast majority of CTE diagnoses occur in individuals with a self-reported or witnessed history of contact-sport-related head injuries or military-related blast exposure (Goldstein et al., 2012; Mez et al., 2017). Accordingly, preclinical efforts to model this disease entity (primarily in rodents) have employed techniques to experimentally deliver repeated impacts to the head (Figure 2). Across laboratories, several variations in the force, frequency, and total number of impacts in such models of CTE exist. In general, most employ a week-long exposure of daily impacts (for a total of 7 exposures, Kondo et al., 2015; Pozdnyakov et al., 2019). A number of procedures have been developed to induce TBI via compressive, focal, or rotational forces. One common method of inducing focal TBI involves stereotaxically delivering a focal impact of precise velocity, depth, and duration to a head-fixed rodent subject. rmTBI mouse models have typically utilized an impact velocity of 3–5 m/s, penetrate the cortical surface by 1–2 mm, and remain engaged with the cortex (“dwell time”) for around 150 ms.

**FIGURE 2:** Two main approaches utilized preclinically to apply standardized and precise trauma to rodents include the stereotaxic approach (left) where a head-restrained rodent receives a vertically oriented impact of a specific velocity, force, and dwell time. More recently, to more closely model blast and other accelerative forces, a standardized rotational impact can be applied (right) by restraining the body and *not* the head, resulting in angular acceleration of the head along either the mediolateral axis (when applied laterally (Goldstein et al., 2012; Logsdon et al., 2017; Chen M. et al., 2018) or along the anteroposterior axis [when applied vertically (Namjoshi et al., 2014)].

This approach does have drawbacks: secondary injuries such as cranial fracture or intracranial hemorrhage do occur at some measurable rate (Kinder et al., 2019). Additionally, stereotaxic impact may have limited translational relevance, since most clinically significant forms of TBI in humans are induced by sudden changes in rotational acceleration. In order to replicate such TBIs, one group employed a gas-driven apparatus to accelerate the head laterally; these mice displayed neuropathological changes resembling CTE including tau phosphorylation, microvascular damage, and perivascular neuroinflammation, without skull fracture or hemorrhage (Tagge et al., 2018). Military personnel are likely to develop CTE through compressive waves via blast exposure. The use of pressure forces can be modeled in a compressed gas blast tube that induces accelerative forces equivalent to 5.8 kg of trinitrotoluene (TNT) at a distance of 5.5 m. In one study, a single blast to 2.5-month-old mice was sufficient to cause long-term vasculopathy, phosphorylated tauopathy, neuroinflammation, and cognitive deficits without cranial damage (Goldstein et al., 2012).

While the more nuanced aspects of CTE-related cellular and molecular derangements remain an active area of research, most agree that a valid preclinical model of CTE should demonstrate evidence of a phosphorylated tauopathy in response to rmTBI. In this regard, insights into CTE pathophysiology may be borrowed from transgenic Alzheimer’s disease models such as TauP301L and 3xTg-AD, with the caveat that these mice develop amyloid and tau pathology even in the absence of rmTBI (Risling et al., 2019). Other models such as transgenic hTau (Morin et al., 2018) or Tgh/Tau (Rubenstein et al., 2019) express human tau gene rather than rodent tau. Such models, when combined with trauma, may better emulate human neurodegeneration because they express all six tau isoforms found in human CTE (Rubenstein et al., 2019). Mice devoid of tau are protected from the long-term changes in exploration and motor coordination following a single fluid percussion injury (Tan et al., 2020): whether these mice may be protected from the effects of rmTBI remains to be defined.

The severity of CTE is dependent on both magnitude and frequency of rmTBI. Many CTE models (Kondo et al., 2015; Pozdnyakov et al., 2019; Rubenstein et al., 2019) induce 5–10 concussive TBIs over a period of a week. While practical in a laboratory setting, this methodology may not be translationally accurate as most reported cases of human CTE occur in individuals with *years* of participation in a contact sport and include individuals who have only received sub-concussive impacts (Sundman et al., 2015). Future studies may more accurately represent sport-related CTE cases by decreasing the magnitude and increasing the frequency and duration of impacts in animal models. One case study suggested that a single severe TBI caused p-tauopathy and neuronal degeneration in secondary affected brain regions, but without the presence of other CTE-associated biomarkers like TDP-45 and alpha-synuclein (Okamura et al., 2019). Importantly, one blast model found that head immobilization during blast exposure did not lead to behavioral deficits, indicating a link between accelerative forces and the development of behavioral symptoms found in mTBI (Goldstein et al., 2012). This finding further suggests that stereotaxic models of TBI may lack clinical relevance.

Anatomical and physiological differences between rodents and humans may also limit current preclinical models. Computational modeling suggests that TBI most directly strains deep sulci (Ghajari et al., 2017), where tau is known to accumulate in CTE (McKee et al., 2016). Rodents do not have sulci, suggesting that preclinical studies could benefit from a higher organism. Recently, pigs have been suggested as a model organism for TBI studies as their cortical surfaces are gyrated and are closer to human brains in size (Kinder et al., 2019). One study applied rmTBI induced by rotational acceleration apparatus and demonstrated evidence of the accumulation of amyloid beta and tau (Chen et al., 2004).

## Immunotherapy

Monoclonal antibody therapy is one of the most promising strategies for combating CTE. Tau accumulation is perhaps the most prominent feature of CTE and thus represents the most intuitive target for antibody therapeutic intervention. Given phosphorylated tau’s strong intraneuronal localization in CTE, one could reason that an intracellular-acting antibody may be more potent in combating tauopathy (Sigurdsson, 2018). However, intracellular translocation of mAbs is challenging and highly dependent on receptor affinity and charge (Sigurdsson, 2018; Katsinelos et al., 2019). Studies have suggested that tau pathology occurs through extracellular mechanisms (Le et al., 2012; Walker et al., 2013); thus, an antibody that acts extracellularly or merely blocks neuronal p-tau import (Nobuhara et al., 2017) may be a feasible alternative. Ideally, effective mAB immunotherapies would preferentially target pathogenic forms of tau protein (Rosenmann, 2013), since tau has an important native role in promoting microtubule transport assembly (Nakamura et al., 2012) and axonal transport (Morris et al., 2011). Similar concerns have been raised over the use of tau-lowering antisense oligonucleotides (ASOs, Jadhav et al., 2019). At least in mice, homozygous deletions of tau do not appear to compromise survival or reproductive fitness but do lead to subtle deficits in standardized measures of learning, memory and anxiety (Gonçalves et al., 2020).

In addition to phosphorylation, one early hallmark of tau pathology is its *trans* to *cis* isomerization. Recent work studying the prolyl isomerase *Pin1* in AD has demonstrated isoform-specific properties of tau that may drive tauopathy (Lu and Zhou, 2007). Generally, tau is actively converted from its *cis* to *trans* isoform via Pin1 but may revert to *cis* tau under stress or hypoxic conditions (Kondo et al., 2015). Unlike *trans* tau, the pathological *cis* tau variant does not associate with microtubules and leads to “*cis-*tauosis” throughout the brain (Kondo et al., 2015). Indeed, *cis-*tau was found to be the prominent isoform found in human CTE brains. Isoform-specific antibodies thus represent one viable way to selectively target pathogenic forms of tau. *cis* phosphorylated tau antibodies with no cross reactivity to *trans* tau or non-phosphorylated tau have been utilized to prevent stress-induced *cis-*tauosis *in vitro*. Additionally, a *cis-*tau-directed mAB prevented TBI-induced cis-tauosis and rescued TBI-dependent behavioral risk-taking behavior in mice (Kondo et al., 2015).

A number of factors impede the use of antibodies to prevent tauopathy in humans. In particular, antibodies must efficiently cross the blood–brain barrier. Antibodies must also be humanized in order to prevent direct attack of antibodies by the human immune system (Congdon et al., 2019). Given that most pathological tau is intracellularly localized, human chimerization of tau antibodies has been shown to alter charge and binding ultimately reducing efficiency (Congdon et al., 2019). While no clinical trials exist specifically for CTE, there are at least half a dozen clinical trials exploring the therapeutic effects of various tau antibodies on patients affected by AD (Sigurdsson, 2018), any of which may address the tauopathy of CTE if they showed success in AD.

Blood–brain barrier (BBB) permeability is one of the main factors limiting the efficacy of antibody treatment in CTE and other neurological diseases. Recent advances in ultrasound technology may be used to aid immune response or drug delivery across the BBB. Unilateral focused ultrasound (FUS) has been a candidate method used to increase BBB permeability by producing transient openings in endothelial tight junctions (Hynynen et al., 2001; Sheikov et al., 2004). Recently, preformed microbubbles have been injected in conjunction with FUS to decrease side effects leading to safe *in vivo* transfer of antibodies and other therapeutics across the BBB (Jordão et al., 2010; Samiotaki et al., 2015). In an AD model, FUS has been shown to assist delivery of amyloid beta antibody delivery (Jordão et al., 2010). In conjunction with FUS, *cis* p-tau mAB may address tauopathy in CTE models. Surprisingly, FUS may reduce tau even in the absence of pharmacological intervention (Karakatsani et al., 2019). While the mechanisms explaining this phenomenon are poorly understood, one hypothesis suggests that increased BBB permeability may enhance anti-p-tau microglial activity surrounding the processes of CA1 pyramidal neurons (Karakatsani et al., 2019). Low-intensity pulsed ultrasound (LIPUS), an additional technique that has shown preclinical success in both TBI (Li et al., 2017; Chen C.-M. et al., 2018) and AD (Lin et al., 2015), has recently been proposed as a non-invasive treatment for CTE (Tsai, 2020). LIPUS treatment in an AD rat model produced significant improvements in a number of CTE-related indices including beta-amyloid formation, acetylcholinesterase, and memory loss (Lin et al., 2015).

## Kinase Inhibitors

The primary mechanism of conversion from functional to pathogenic tau is hyperphosphorylation (Miao et al., 2019). Phosphorylation at various sites leads to tau dissociation from microtubules and the formation of neurofibrillary tangles (NFTs). Tau hyperphosphorylation occurs at eight or more sites, each of which could be therapeutically targeted via kinase inhibition. The most critical phosphorylation sites are Thr175 and Thr231 (Lin et al., 2007; Kondo et al., 2015; Moszczynski et al., 2018; Katsumoto et al., 2019). Tau hyperphosphorylation activates glycogen synthase 3 beta (GSK-3B) which results in further tau threonine phosphorylation and formation of NFTs. GSK-3B is a logical target for therapeutic intervention not only because of tau phosphorylation but also because of its role in downregulating antioxidant defenses. GSK-3B inhibits the transcription factor Nrf2 required for the transcription of heme oxygenase-1, capable of metabolizing reactive oxygen species (ROS) associated with a variety of neurodegenerative processes (Rojo et al., 2008). Thus, potent and selective GSK-3B inhibitors have been explored as a treatment for CTE (Kabadi et al., 2012). One such inhibitor, dimethyl fumarate (DMF), has shown preclinical success in a non-TBI-based model of tauopathy. DMF administration successfully activated the Nrf2 pathway and prevented p-tau-dependent astrogliosis and microgliosis (Cuadrado et al., 2017). In addition to DMF, most studies of GSK-3B inhibition have focused on lithium treatment. Lithium directly inhibits GSK-3B by binding to its magnesium-binding site and also indirectly inhibits GSK-3B activity by activating upstream GSK-3B inhibitors phosphatidylinositol 3-kinase (PI3K) and protein kinase B (AKT) (Chalecka-Franaszek and Chuang, 1999; Leeds et al., 2014). In multiple *in vitro* and *in vivo* models, lithium treatment has been shown to ameliorate tau phosphorylation, microglial activation, neuronal death, amyloid beta formation, and neuroinflammation while preserving cognitive function and BBB integrity (Dash et al., 2011; Ekici et al., 2014; Zhu et al., 2010; Yu et al., 2012).

Other kinases such as cyclin-dependent kinases (Cdks) are also involved in pathological tau hyperphosphorylation. The potent CDK inhibitor roscovitine has been studied in models of TBI and demonstrated attenuation of neurodegeneration in a model of controlled cortical impact in mice (Kabadi et al., 2012). Combining multiple kinase-targeting therapies may provide a synergistic effect; one study found that a combination of both lithium and roscovitine better prevented tau pathology in response to rmTBI than a single kinase inhibitor alone (Rubenstein et al., 2019). These results correlated with a significant reduction of phosphorylated tau both in blood serum and cortex after rmTBI and rescued impairments in motor function and spatial memory.

## Anti-inflammation

Beyond tau hyperphosphorylation, the progression of CTE is thought to include a complex cascade of secondary inflammatory and metabolic changes that may also represent potential targets for therapeutic intervention (Kulbe and Hall, 2017). Ionic imbalances and dysfunctional neurotransmitter release that occur following neuronal injury result in microglial and astrocyte recruitment. TBI itself causes an increase in BBB barrier permeability, which can lead to the infiltration of larger, potentially toxic molecules into the parenchyma (Karve et al., 2016), further amplifying neuroinflammation. Microglia and astrocytes secrete inflammatory cytokines and chemokines that can have a combination of neurotoxic or neuroprotective effects (Kulbe and Hall, 2017). Microglia are felt to generally have a protective role in TBI, but chronic microglial activation releases microparticles associated with neurodegeneration into circulation. These extracellular vesicles activate pro-inflammatory mediators such as IL-1B, TNF-a, CCL2, IL-6, and NOS2 (Kumar et al., 2017). Activation of voltage-gated channels following primary neuronal injury also leads to an influx of calcium ions, setting off a complex cascade of neurodegenerative processes (Weber, 2012). In order to maintain calcium homeostasis, mitochondria must release intracellular calcium stores at the expense of cellular respiration. Such mitochondrial compensation results in the formation of highly neurotoxic oxidative species that induce DNA damage, mitochondrial death, and apoptosis (Kulbe and Hall, 2017).

The production of reactive oxidative species and mitochondrial stress likely plays a key role in driving neuronal ischemia in CTE (Pozdnyakov et al., 2019). These pathways may be halted through administration of mitochondrial-protective pyrimidine derivatives. Intraperitoneal administration of one such pyrimidine derivative abbreviated “OCH” (4-{2-[2-(3,4-dimethoxyphenyl)-vinyl]-6-ethyl-4-oxo-5-phenyl-4H-pyrimidine-1-Il}benzsulfamide) during a rmTBI rat model provided significant preservation of mitochondrial respiration and glycolytic activity. Additionally, OCH-treated rats displayed a reduction in CTE-associated markers GFAP, NSE, S100 beta, and beta-amyloid, together with improvements in sensorimotor control assessed through a beam-walking task (Pozdnyakov et al., 2019). Another promising strategy to control neuroinflammation following rmTBI may be through modulation of arachidonic acid metabolism. The role of this pathway in tauopathies is not totally understood; one study found that arachidonic acid administration delays neurodegeneration in AD (Schaeffer et al., 2009), whereas other studies have suggested that arachidonic acid is a central driver of neurodegeneration (Amtul et al., 2012). Recent rmTBI models focused on a product of arachidonic acid metabolism, the endocannabinoid 2-arachidonoylglycerol (2-AG). Inhibiting the enzyme monoacylglycerol lipase (MAGL) preserved 2-AG levels, leading to a reduction in proinflammatory cytokines, amyloid-beta precursors, and astrocyte reactivity (Panikashvili et al., 2006). Encouragingly, inhibition of this pathway via MAGL inhibitor JZL184 in a rodent model of rmTBI also led to corresponding attenuation of neurodegeneration, tau phosphorylation, and beta-amyloid synthesis (Zhang et al., 2015).

## Conclusion

Sadly, despite increasing recognition among athletes and military personnel, there are currently no available treatments for CTE or practical clinical diagnostic markers to identify at-risk individuals. Fortunately, with a detailed neuropathological description from postmortem samples combined with preclinical models that have been inspired by the Alzheimer’s field, we are closer to obtaining a comprehensive pathophysiological understanding of CTE. Like AD, CTE is a progressive neurodegenerative disease that appears to propagate via tau phosphorylation and subsequent aggregation into neurofibrillary tangles. At the same time, trauma-induced changes in circuit function may borrow from prior research in severe traumatic brain injury. While research on these related conditions may shed light on CTE pathology, it also warns of potential pitfalls. In particular, both AD and severe TBI (Stein, 2015) have suffered numerous failed clinical trials in spite of enormous preclinical successes. In order to avoid losing candidate therapies in translation, CTE research must not only address fundamental differences between human patients and animal models but also ensure the development of robust preclinical CTE models that may continue to build on pathomechanistic insights and candidate treatments. Currently, some preclinical models of CTE fail to demonstrate tau pathology (Pozdnyakov et al., 2019) or attain it without TBI (Morin et al., 2018). A variety of reliable models may be useful to encapsulate the heterogeneous nature of TBIs. However, these models should focus on delivering multiple impacts that generate accelerative forces to the head in place of or in addition to stereotaxic impact. The field would also benefit from a systematic evaluation of trauma frequency (daily vs. weekly, etc.) and assessments at more delayed time points. Unbiased proteomic/phosphoproteomic approaches may provide a more comprehensive picture of “kinome” changes following rmTBI and may aid in the development and screening of mABs. EEG studies may also be essential to explore whether cognitive phenotypes seen in these CTE models may be associated with spontaneous seizures.

Perhaps the most intuitive way to halt the progress of CTE is to inhibit processes directly affecting tau phosphorylation and aggregation. Given tau’s multiple physiological functions, therapies must selectively inhibit formation and spreading of pathogenic tau. A profile of kinases directly phosphorylating tau in CTE has been developed and opened the door to a number of kinase inhibitors such as roscovitine and lithium which have shown promising preclinical results. The recent finding that tau is converted from a functional *trans* to pathogenic *cis* form has driven the development of isoform-specific phosphorylated tau monoclonal antibodies. The use of immunotherapy is one of the most promising strategies to treat CTE and other neurodegenerative diseases but suffers from poor translational efficiency. Techniques such as FUS/LIPUS may be used in conjunction with antibody treatment to improve the delivery of *cis* p-tau antibodies and immune agents across the blood–brain barrier.

As these candidate therapies move forward to clinical phases, researchers should note the failure of dementia research to produce successful clinical trials (Gauthier et al., 2016). Why do so many drugs showing significant preclinical success fail in translation, and how can this be avoided with CTE research? One consideration is the time of drug administration (Anderson et al., 2017); therapies may be administered when the underlying pathology is too advanced for the candidate drug to work effectively. While the temporal characteristics of CTE pathology are not totally understood, symptoms may not appear until decades after rmTBI. Like CTE, AD pathology likely develops for years before symptoms appear, yet most failed AD clinical trials have selected patients in the middle to late stages of the disease. Fortunately, since CTE has a more concretely defined etiology and affects specific demographics, future treatments for CTE may take the form of a preventative/prophylactic medication applied to at-risk individuals during or even before participation in contact sports.

## Author Contributions

PB and VK played significant roles in the initial manuscript drafts and subsequent revisions.

## Conflict of Interest

The authors declare that the research was conducted in the absence of any commercial or financial relationships that could be construed as a potential conflict of interest.
